RETRACTED

# Prediction Model of Piano Collective Class Teaching and Learning Effect Based on Deep Learning

**DOI:** 10.1155/2022/2572372

**Published:** 2022-07-18

**Authors:** Xiaoyue Zhu

**Affiliations:** Shanghai Normal University TIANHUA College, Shanghai 201815, China

## Abstract

This paper proposes a prediction model of piano collective class teaching and learning effect based on DL network in order to realise the precise prediction and evaluation of piano collective class instructional effect and promote the improvement of piano collective class instructional quality. The idea of an instructional assessment index is quantified in this paper using specific data as its input and educational impact as its output. In parallel, several training networks are established to correspond to the first-level evaluation indexes, and the input samples are normalised. Finally, MATLAB performs the empirical research. According to the findings, this method's prediction accuracy can reach 94.41 percent, which is about 10.22 percent higher than that of conventional methods. This prediction model is somewhat realistic and feasible. When used to predict and assess instructional quality, this method not only eliminates the subjectivity of experts in the evaluation process but also yields satisfactory evaluation outcomes and has a broad range of applications. According to the model's predictions and evaluation findings in this paper, appropriate teachers can better understand the drawbacks of the collective class model, focus on some important aspects of teaching activities, and then enhance instructional methods and effects.

## 1. Introduction

With the rapid pace of educational reform and development, numerous instructional methods have been continuously improved and perfected, new models and theories suitable for curriculum teaching reform and development have been developed, and classroom teaching reform research has been conducted in full force [1]. For students majoring in music education, piano is a fundamental and required course. For many professional students, piano lessons are crucial. For instance, in order to fulfil the requirements for teaching, students who will eventually be involved in preschool education or other levels of music teaching must master a specific set of piano skills [2]. The reform and advancement of music education in normal universities, as well as the theoretical inspiration and enlightenment of foreign piano teaching models, served as the foundation for the development of piano collective class instruction in these institutions. In typical universities, piano is a crucial course, and group instruction is a common practise that is unavoidable given the growing student population. Piano instruction in typical universities has quickly evolved to include group piano lessons. The issues with piano teachers' “one-on-one” workload, small lecture spaces, and repetitive lectures have been resolved by group piano lessons [3]. This teaching approach can be described as sophisticated and practical, and its application also has higher scientific requirements. Piano collective class, however, is a new course compared to the conventional piano “one-to-one” teaching mode, and as such, it will inevitably run into various issues and conundrums during its implementation. A topic worth studying is how to increase teaching effectiveness because collective teaching must deal with a large number of students. Piano collective class teaching has in fact opened up a new and effective way for piano teaching in normal universities, which has drawn more and more attention from teachers and students majoring in music education in normal universities. This has been done in order to implement quality-oriented education and speed up the training of talents in basic music education.

RETRACTED

This paper presents a prediction model of the teaching and learning effect of piano collective class based on DL (Deep learning) [4–6] network in order to realise the accurate prediction and evaluation of piano collective class instructional effect and promote the improvement of piano collective class instructional quality. Currently, many straightforward methods are used to assess the quality of instruction in colleges and universities, including the absolute evaluation method, relative evaluation method, rating method, comment method, realistic method, and comprehensive scoring method. It is difficult for the results of these methods to accurately reflect the quality of the instruction because they are either overly subjective or they omit the nonlinear relationship between each evaluation index and the instructional effect when evaluating the instructional effect. Additionally, it is challenging to express the evaluation result of the quality of instruction using a linear mathematical formula because there are numerous factors that influence the evaluation and all of the factors are interrelated. The NN (Neural Network) [7, 8] is a massively parallel processing-based nonlinear adaptive dynamic system. It mimics the information-processing mechanisms of the brain at various levels and has the capacity to learn, remember, compute, and use intelligent processing [9]. The DL network is an extension of the NN, which has excellent feature learning capabilities. The restored data characteristics can be used to create effective data visualisations and classifications. Essentially, DL is a type of dynamic information processing system made up of numerous information processing units connected in a variety of ways. This paper, which is based on the DL method, is concerned with the prediction of piano collective class teaching and learning effect.

RETRACTED

The contributions of this paper are summarized as follows. (1) In this paper, DL technology is used to predict the teaching and learning effects of piano collective classes, and a system of evaluation indexes for the calibre of piano collective class instruction is developed. A rich basic data set for instructional assessment has been created on this basis through the evaluation of teaching experts, teachers' peers, and students. According to the research, this model can avoid subjectivity in the process of expert prediction and offers a novel idea and approach for the prediction and assessment of the overall quality of piano instruction. (2) The program's functional structure design, database design, and primary technical issues are all thoroughly discussed. On this foundation, it discusses the methods for statistical result analysis and processing, briefly describes the recording, collection, preservation, and updating of tracking data, and implements the software system for this model in real-world settings. The results of the system's operation evaluation indicate that the evaluation findings and analysis data can serve as a point of reference for the assessment of the effectiveness of group piano instruction and supporting decision-making.

## 2. Related Work

Bhandari et al. used the adaptive and self-learning principles of BPNN (Back propagation neural network) for instructional quality evaluation, and proposed an NN-based instructional quality evaluation model structure and an improved BP network learning algorithm [10]. Donlan and Byrne pointed out that the introduction of evaluation methods in the teaching of piano group lessons will help teachers to fully understand the whole process of teaching, adjust teaching strategies in time, improve students' self-confidence, and stimulate their inner learning motivation; thus realizing piano learning as soon as possible autonomy and the formation of quality education [11, 12]. Capella-Peris et al. pointed out that the diversified instructional methods, interactive teaching process, and comprehensive teaching content of piano group lessons in normal normal schools are conducive to cultivating students' keyboard performance application, cooperation, performance, and creativity; Comprehensive quality of music [13]. Based on the simulation experiment of the instructional assessment model of BPNN, Nashon and Anderson constructed a set of teacher instructional assessment system with this evaluation model as the core [14]. The system mainly includes functional modules such as online evaluation of instructional quality, management of evaluation results, and comprehensive information query. Shang believes that the piano group class solves the problem of “one-to-one” piano teachers' heavy workload and repeated teaching to a certain extent. Therefore, this instructional method is a combination of advanced nature and practicality [15]. Liang pointed out that the application of NN model in instructional assessment depends on the user's mastery of NN theory, and needs to master some skills of data processing. Training NN through reasonable sorting of known data can make the network training faster and more accurate [16]. On the basis of studying the characteristics of network-based teacher instructional assessment, Sciandra et al. analyzed the basic theories and methods of traditional college instructional assessment. By combing the theory and reflecting on time to form an evaluation strategy, a teacher instructional assessment model based on evaluation files is constructed [17].

RETRACTED

This paper presents a fresh research angle and approach based on studies on the teaching and learning effects of group piano lessons in pertinent literature. This study, which is based on the DL method, aims to predict the teaching and learning outcomes for piano collective classes. Discussions of the program's primary technical issues, database design, and functional structure are in-depth. On this foundation, it briefly describes the recording, collection, preservation, and update of tracking data, discusses the methods for processing statistical results, and implements the software system for this model in real-world settings. According to the study, it can offer some workable methods for teaching piano to a group of students as well as some useful resources for teachers in related fields.

## 3. Methodology

### 3.1. Related Theoretical and Technical Basis

In order to speed up the training of talents in basic music education, piano collective class teaching has indeed opened up a new way for piano teaching in normal universities, which has attracted more and more attention from teachers and students of music education major in normal universities. As far as higher art education is concerned under the new situation, the instructional method of piano collective class is superior to the traditional instructional method. However, there are some drawbacks in the current teaching mode of piano collective class, which leads to the fact that the instructional effectiveness is not as good as expected. Therefore, it is necessary to innovate and improve teaching activities, and constantly improve the effectiveness of collective piano lessons [18]. To achieve this, it is necessary to effectively and accurately predict and evaluate the instructional quality of collective piano lessons. Predicting and evaluating instructional quality is an important link in teaching management, and its fundamental purpose is to master teachers' actual teaching ability and level and encourage and promote teachers to follow the teaching laws and principles, improve the instructional quality, cultivate qualified talents, and optimize the teaching staff according to the requirements of training objectives. Usually, the evaluation based on experts' experience leads to the subjective randomness of the evaluation, and there is a certain error between the evaluation result and the actual value; it is difficult to evaluate the results of some indexes accurately by traditional methods, and the calculation is complicated and the solution is tedious. These algorithms also lack self-learning ability. As a new instructional assessment model, the evaluation model of piano collective class has the characteristics of development, diversification, openness, and comprehensiveness, which can weaken the screening and selection function and strengthen and improve the incentive function in teaching. DL has a strong feature learning ability, the learned features can restore the characteristics of data, and it has a good visualization and data classification effect [19]. DL system has unique functions in dealing with all kinds of fuzzy, random, large-volume, dynamic, and low-precision information [20]. The DL model is shown in Figure 1.

RETRACTED

BPNN is a feedforward network composed of multilayer neurons. The novelty of BPNN is that it can model the nonlinear process without knowing the reason of data generation, and it has the characteristics of nonlinear mapping, learning classification and real-time optimization [21]. Requirement analysis is the purpose and foundation of software design and development, which explains the reasons of software development. The most fundamental thing is to know the specific needs of customers, which is also applicable to this instructional assessment system. Therefore, the development of this system also needs to meet the basic needs of the evaluation subjects. The system built in this paper should have the following performances: (1) The system is easy to use and easy to maintain. (2) Openness and expandability of system. (3) The standardization and advancement of system. (4) High response speed of the system. According to the hierarchical method, this paper establishes the evaluation index system for the object to be measured. First, the top index is defined as the whole, and then the whole is subdivided into several subitems such as teaching management, teaching attitude, and other first-level indicators. The first-level indicators are divided into a plurality of second-level indicators. You can also continue to subdivide according to actual requirements. All the participating projects constitute an index system with hierarchical structure. The evaluation index system of this paper is shown in Table 1.

RETRACTED

NN training, NN evaluation, and sample data maintenance are all parts of the NN evaluation module. Its job is to finish managing and educating instructional assessment data as well as forecasting and assessing instructional quality based on it. The sending and receiving portions of the window should be real-time on the same day so they can reflect the status of being inspected and sent right away. As this system is a predictive evaluation management system, the basic information should be updated at any time in accordance with the school construction, and the comments submitted by the administrators can be updated at any time. Through a firewall management programme, the system administrator creates, updates, and loads the security rules firewall. The system's primary job is to analyse and fit the results of instructional assessment, which is broken down into four components, including NN and sample data preprocessing. In order to confirm students' innate cognitive process and cognitive deficiency in the process of learning piano, the new teaching intervention method can help teachers use and create a simple dynamic evaluation method flexibly in accordance with the realities of teaching and evaluation as well as the characteristics of piano teaching and performance. The development of a system for monitoring and forecasting instructional quality in this paper is crucial for enhancing instructional quality and ensuring instructional effect.

### 3.2. Construction of Prediction Model of Collective Piano Teaching and Learning Effect

The NN-based prediction system of piano collective class teaching and learning effect is divided into three key steps: (1) It is necessary to prepare the data that meets the requirements of the index, and take the qualified data as the input training samples of the network, then correctly construct the BPNN and train the network. (2) Evaluate the training network established in the first step to evaluate the actual effect of network training. (3) Get the training effect of the network, and then get a real and effective NN evaluation model. In this paper, the network structure of single output layer will be selected, then the network output value is the comprehensive evaluation value of instructional quality. For the nonlinear function approximation problem network, the transfer function of hidden layer neurons can choose S-type tangent function, and the transfer function of output neurons can choose S-type logarithmic function, and the output is between 0 and 1. At this time, the network can realise any nonlinear mapping from input to output. The forward propagation and backward propagation of BPNN alternate with each other, which can be regarded as a process of “memory training.” Because the original instructional assessment result data is greatly influenced by the evaluators, the original evaluation data must do some preliminary data processing to interfere with the evaluation; otherwise it will affect the prediction result of NN, and also affect the learning speed and calculation accuracy of the algorithm. The function of instructional quality prediction is the core function of this system. Through this function, teachers' instructional quality can be evaluated objectively and fairly. Users who participate in the instructional quality evaluation activities include students, teachers, teaching management experts, system administrators, and other roles. The network architecture and algorithm training process are shown in Figure 2.

RETRACTED

The activities involved in instructional assessment can be broken down into the following categories: gathering and initialising teaching raw data, building an evaluation system, putting instructional assessment into practise, processing and producing evaluation results, and gathering evaluation information. In this study, the perceptron's connection weight distribution and network structure are modified using the adaptive learning algorithm to get closer to the desired input-to-output mapping. When the network is stable, the structure of network preservation and the distribution of weights will reflect the expertise and experience of industry experts in resolving this issue. The original teaching-related data should be preprocessed before the NN algorithm training operation, and the effectiveness and outcomes of the evaluation algorithm will be directly impacted by the quality of the preprocessing. Consequently, normalising the original data should come first. The input vector for a three-layer BPNN is

(1) $$\begin{array}{c} X={\left(x_{1},x_{2},x_{3},\ldots ,x_{i},\ldots ,x_{n}\right)}^{T}. \end{array}$$

Implicit layer output vector is

(2) $$\begin{array}{c} Y={\left(y_{1},y_{2},y_{3},\ldots ,y_{j},\ldots ,y_{m}\right)}^{T}. \end{array}$$

The output vector of the output layer is

(3) $$\begin{array}{c} O={\left(o_{1},o_{2},o_{3},\ldots ,o_{k},\ldots ,o_{l}\right)}^{T}. \end{array}$$

The weight matrix between the input layer and the hidden layer is

(4) $$\begin{array}{c} V={\left(V_{1},V_{2},V_{3},\ldots ,V_{j},\ldots ,V_{m}\right)}^{T}. \end{array}$$

The number of hidden units is directly related to the requirements of the problem and the number of input and output units. Too many hidden layer units will lead to problems such as too long NN training time, difficult error control, and poor fault tolerance. In the process of NN application, there are generally three ways to determine hidden layer nodes as follows:

(5) $$\begin{array}{c} m=\sqrt{n+1}+\alpha , \end{array}$$

(6) $$\begin{array}{c} m=\log\;2^{n}, \end{array}$$

(7) $$\begin{array}{c} m=\sqrt{n1}. \end{array}$$

Among them, *m* is the number of hidden layer nodes; *n* is the number of input layer nodes; 1 is the number of output layer nodes; *α* is a constant between 1 and 10. This paper chooses formula (6) to determine the number of hidden layer nodes. Let the weight vector be

(8) $$\begin{array}{c} W=\left(w_{1},w_{2},w_{3},\ldots ,w_{n}\right),\\ w_{i}\left(i=1,2,3,\ldots ,n\right),\\ x_{i}\left(i=1,2,3,\ldots ,n\right). \end{array}$$

Among them, *w*_*i*_ represents the importance of factor *x*_*i*_, which satisfies

(9) $$\begin{array}{c} \sum_{i=1}^{n}w_{i}=1,0\leq w_{i}\leq 1. \end{array}$$

The cumulative error is calculated using the following formula: Gradient descent is used to solve the approximation problem of NN, which is briefly explained. First, take *X*=[*x*_1_, *x*_2_, *x*_3_,…, *x*_*n*_] as the input vector of the training network; take *H*=[*y*_1_, *y*_2_, *y*_3_,…, *y*_*j*_] as the radial vector of the training network, then the Gaussian function formula is

(10) $$\begin{array}{c} y_{j}=\exp\left(-\frac{{\left\|X-C_{j}\right\|}^{2}}{2b_{j}^{2}}\right),j=1,2,3,\ldots ,m, \end{array}$$

where *C*_*j*_=[*c*_1*j*_, *c*_2*j*_, *c*_3*j*_,…, *c*_*ij*_,…, *c*_*nj*_] is the center vector of the *j* th node of the neural training network; *B*=[*b*_1_, *b*_2_, *b*_3_,…, *b*_*m*_] is the base width vector; *b*_*j*_ is the base width parameter of the node *j*. And *b*_*j*_ > 0. *W*=[*w*_1_, *w*_2_, *w*_3_,…, *w*_*m*_] is the weight vector of the network.

RETRACTED

When the parameters are optimized, according to the characteristics to be tested, after learning the deep belief network model with trained model parameters, calculate the probability that this characteristic belongs to the online instructional quality scores of colleges and universities, and select the quality score with the highest probability as the output result. In this system, according to different users' query authority, administrators/experts can query all information, teachers can query information about classes, students, and personal evaluation results; students can view personal information and evaluation information of teachers who have been evaluated. This model has the advantages of high efficiency and precision and can ensure the objectivity of the evaluation results.

## 4. Result Analysis and Discussion

Software should be tested once it has completed all of its development. The aim of testing, however, is to identify flaws. A test that discovers errors that have not yet been discovered is considered successful. By testing a system, we can identify any issues with it, determine whether the system software we designed and developed can satisfy user needs, and determine whether the software satisfies quality standards. The full definition of software testing is: a thorough process of identifying programme flaws and confirming that the system's performance and function adhere to the specifications, using appropriate technical tools and programmes that are executed in a complex control system environment. In this study, the software is put to the test in order to identify and address any issues that may be present, ultimately enhancing the software's dependability and quality. Software compatibility and nonfunctionality should also be tested during testing, and these should be tested in various browser environments in addition to testing software functions. The aforementioned instructional quality prediction system is found using NN in this chapter. The learning rate is 0.9, and the input layer has 36 neurons, the hidden layer has 10 neurons, and the output layer has one. The normalised data are used as training samples for an NN model. MATLAB training software is used, with a target error of 0.001.

The accuracy of data depends on the accuracy of data, that is, the accuracy of final evaluation results should be high, vague evaluation is not allowed, and the accuracy cannot be changed in the process of data transmission. The accuracy of collected data should be consistent with the corresponding output data. The requirement of the accuracy of the input and output data of the software is to accurately evaluate the teaching results, and there should be no vague evaluation, which may include that the accuracy cannot change during transmission. The accuracy of the input data comes from the data accuracy involved in various operations in the user's business process. There will always be some errors between the BP network trained by MATLAB and the exact value. The results obtained in this paper are similar to those of existing network training. MATLAB software provides a powerful Simulink tool that can help adjust various parameters in a specific NN, and it is very convenient to implement. The network training results are shown in Figure 3.

RETRACTED

The output accuracy of the network depends on the number of input training samples. The more training samples are, the closer the predicted value of the output instructional effect is to the actual evaluation value. Data conversion and transmission time: students need to register before instructional assessment, which takes a certain amount of time. Similarly, the calculation of final evaluation results also takes a corresponding amount of time, both of which need to be reduced as much as possible to improve the efficiency of the system. Comparison of operating efficiency of different systems is shown in Figure 4.

In the Simulink environment, the trained NN module is used to simulate network data, and the random number generator is used to generate various input vector groups. These random vectors must be normalised and transformed into the input data of NN by normalisation function in order to make the input vectors conform to the actual meaning of the input data. When testing, it is important to finish formulating test cases in accordance with the requirements of the system application, compile test cases based on the test plan, and simultaneously verify the system specifications and design. To complete the system programme code test and ensure the accuracy of the data of tiny units in the running process, the internal programme test of the system needs to be strengthened. To this end, the unit test methodology is used. All units must be integrated before the test, and the results and functionality of the integrated units must be tested. The prediction errors of different systems are shown in Figure 5.

The experimental results show that the trained model has the accuracy of prediction and can be effectively used to predict the learning effect of collective piano lessons. After the network training is completed, another set of data is used to test it. In this paper, 10 groups of samples were randomly selected, and then the error between the evaluation target value output by NN and the actual evaluation target value was checked. The comparison results are shown in Table 2.

It can be seen from the data in the table that the output value of the instructional quality prediction model established by NN is very close to the real value. That is to say, the model can accurately determine the instructional effect according to each evaluation index. Permission is the permission set by different users to use the system, so that users can set their own conditions within the constraint range of system operation. The comprehensive data query function of the system is the query function that the system provides various information including evaluation data, evaluation results, personal data information, etc. for all kinds of users. Most query operations provide the function of exporting query results. The stability test results of the system are shown in Figure 6.

RETRACTED

It can be seen that the system in this paper can maintain a certain stability even if the sample size is large. Each evaluation standard has its own weight. In this paper, the gradient descent method is used to adjust the weight. The setting of the weight is very important, and the reasonable setting of the weight can make the evaluation result more objective and reasonable. In the process of establishing evaluation index, it is necessary to put forward certain requirements for the setting of weights. In this paper, the openness of NN is introduced, so that the network can freely adjust the weights and thresholds, which can achieve better results. The prediction accuracy of different algorithms is shown in Figure 7.

According to experimental findings, this method's prediction accuracy can reach 94.41 percent, which is about 10.22 percent higher than that of conventional methods. The prediction model can utilise NN's self-learning, self-adaptation, and nonlinear approximation capabilities to calculate the quantitative evaluation while also quantifying the subjective factors in the current evaluation system based on expert ratings. Its calculation efficiency is higher than that of the current evaluation system. The outcomes demonstrate the applicability and dependability of this prediction model.

## 5. Conclusions

It should be noted that the teaching method of the collective class is introduced into the piano course, and its main goal is to alleviate the imbalance of teaching proportion caused by the increase in enrollment, so piano teachers can be partially released from the dilemma of an overwhelming teaching workload caused by the ineffective form of “one-on-one” teaching. We must admit that there are some drawbacks to the collective piano teaching, despite the fact that it has clear benefits for developing students. In order to improve instructional effectiveness when teaching piano in collective classes at regular universities, it is important to have a thorough understanding of some current issues and shortfalls, be aware of the drawbacks of the collective class mode, pay close attention to some crucial teaching activities, and then implement creative reforms from the perspectives of student interest, hierarchical teaching, and piano practise. Predicting and assessing the learning impact of group piano lessons is therefore necessary. This study, which is based on the DL method, aims to predict the teaching and learning outcomes for piano collective classes. This paper has developed a rich basic data set of instructional assessment through the evaluation of teaching experts, teachers' peers, and students. The prediction accuracy of this method, according to experimental results, is as high as 94.41 percent, which is roughly 10.22 percent higher than that of conventional methods. There are some practical and feasible aspects to this prediction model. According to the model's predictions and evaluation findings in this paper, appropriate teachers can better understand the drawbacks of the collective class model by paying attention to some crucial aspects of teaching activities. These teachers can then enhance their teaching strategies and the outcomes of their lessons.

RETRACTED

## Figures and Tables

**Figure 1:** DL model.

**Figure 2:** System network architecture and algorithm training flowchart.

**Figure 3:** Network training results.

**Figure 4:** Comparison of operating efficiency of different systems.

**Figure 5:** Comparison of prediction errors of different systems.

**Figure 6:** Stability test results of the system.

**Figure 7:** Prediction accuracy of different algorithms.

**Table 1:** Evaluation index system.

	Primary index	Secondary index
Evaluation index system	Teaching attitude	Professional ethics
		Seriousness of lesson preparation
		Professionalism
		Teacher quality
	Instructional method	Learning method guidance
		Stimulate students' interest
		Take care of personality differences
	Teaching content	Clear teaching objectives
		Appropriate classroom content
	Teaching ability	Professional knowledge
		Blackboard writing
		Language expression
	Instructional effectiveness	Students' mastery
		Popularity of teachers

**Table 2:** Comparison between NN output value and actual evaluation value.

Sample	Network output value	Actual value
1	7.32	7.29
2	7.66	7.65
3	7.51	7.63
4	6.11	6.07
5	7.25	7.31
6	5.21	5.19
7	7.98	7.94
8	7.78	7.82
9	5.42	5.54
10	8.46	8.51

## Data Availability

The data used to support the findings of this study are available from the corresponding author upon request.
